The article "Healthcare and Scientific Treatment of Knee Osteoarthritis" was retracted in 2023. Reasons: signs of a paper mill; compromised peer review; unreliable results or conclusions.

# Healthcare and Scientific Treatment of Knee Osteoarthritis

**DOI:** 10.1155/2022/5919686

**Published:** 2022-01-28

**Authors:** Huan Wang, Baoan Ma

**Affiliations:** Orthopedics, The Second Affiliated Hospital of the Air Military Force Military Medical University, Xi'an, Shanxi Province 710000, China

## Abstract

Knee osteoarthritis is a chronic degenerative disease companied with chronic knee pain and dysfunction. However, the etiology and pathogenesis of knee osteoarthritis were unclear. Currently, age, diet, trauma, obesity, and inheritance are the main risk factors. The major pathological hallmarks of knee osteoarthritis included subchondral bone sclerosis, articular cartilage degeneration, arthrosynovitis, and osteophyte. With the acceleration of the aging process in China, the treatment of knee arthritis and the methods to improve the quality of life have become the focus of medical staff. Currently, therapies in clinical practice include surgery and nonoperative treatment; however, the clinical effects of different individuals at different stages will still be very different. This article reviews the recent advances in the treatment of knee osteoarthritis from three aspects: nonsurgical treatment, surgical treatment, and modern new medical means.

## 1. Introduction

Knee osteoarthritis (KOA) is a type of chronic degenerative arthritis [1], and its chronic inflammation is characterized by degeneration or loss of articular cartilage, articular margin, and subchondral bone regeneration [2]. However, the etiology and pathogenesis of knee osteoarthritis were unclear. With the acceleration of the aging process in China, the incidence rate of KOA is increasing [3]. The methods of improving the quality of life [4–7] and the living standards of patients become an urgent problem for medical workers. At present, there is still controversy about which intervention is the best method.

Currently therapies in clinical practice include surgery and nonoperative treatment; however, the clinical effects of different individuals at different stages will still be very different. This article reviews the recent advances in the treatment of knee osteoarthritis from three aspects: nonsurgical treatment, surgical treatment, and modern new medical means.

### 1.1. The Etiology and Pathogenesis of KOA

Currently, age, diet, trauma, obesity, and inheritance are the main risk factors [8–10]. The articular cartilage layer is worn out, the biomechanical changes in contact with the subchondral bone, and the loss and reduction of articular fluid with the acceleration of the aging process. In addition, with weight gain, ligament degeneration, relaxation, and muscle weakness, there were obvious degenerative changes in articular cartilage and subchondral bone [11]. Inflammatory cells inside the joint, including macrophages, release inflammatory factors [12–14], accelerate the degradation of articular cartilage, aggravate the inflammation of the synovial joint, and produce early inflammatory pain. As mechanistic research continues, relevant cytokines and signaling pathways involved in developing arthritis are also constantly mined, including TGF-*β*, neural growth factor (NGF), and hypoxia-inducible factor (HIF) [15, 16]. Although the pathogenesis of KOA is still unclear, we have found the key to opening the door, provided a strong basis for better achieving the molecular level of treatment intervention; moreover, we do our best to improve the quality of life.

The article "Healthcare and Scientific Treatment of Knee Osteoarthritis" was retracted in 2023. Reasons: signs of a paper mill; compromised peer review; unreliable results or conclusions.

## 2. Conservative Treatment of Knee Osteoarthritis

At present, there are many conservative treatments methods for primary KOA in middle-aged; although it can play a role in improving and delay progressing of the disease, there are some elderly patients with poor curative effects.

### 2.1. Nondrug Treatment

In the early stage of KOA, patients had no obvious symptoms, and it did not impact on work and life; patients can take actions like self-management, prevention to improve the function of the knee joint and improve the quality of life, moreover, delaying and changing the pathological process of osteoarthritis.

#### 2.1.1. Health Education and Health Promotion

Through health education, patients could cultivate a healthy lifestyle including avoiding wind chill, weight loss, and reasonable physical exercise, avoiding such as climbing, squatting, and long-distance running. Effective emotional counseling to guide patients is particularly important [17, 18]. The effect of weight on the knee is of unique importance, and weight loss makes patients the most benefited from interventions [19–21]. Hacken et al. [21] found that weight loss was a reliable method to reduce pain and stiffness and improve function during the five-year follow-up. However, weight control cannot be achieved by dieting. Pay special attention to the intake of fruits and vegetables, such as blueberries, raspberries, and grass pomegranates, which can reduce arthritis pain [22].

#### 2.1.2. Exercise Therapy

Chronic knee pain seriously influences normal life of patients. Patients often have difficulty choosing between restricted activity and appropriate and reasonable exercise. The lack of formal therapeutic rehabilitation training is often the factor of causing the further development of knee osteoarthritis [23]. The clinical effect of muscle strength training is remarkable, which can effectively relieve pain in patients and promote the recovery of knee function [24, 25]. At the same time, Dong et al. found that water sport was comparable to land exercise in the therapeutic effect, but patients had better compliance and satisfaction [26]. Tai Chi in traditional medicine in China also has a good curative effect [27].

The article "Healthcare and Scientific Treatment of Knee Osteoarthritis" was retracted in 2023. Reasons: signs of a paper mill; compromised peer review; unreliable results or conclusions.

#### 2.1.3. Physical Therapy

There are many current physical treatments, such as electromagnetic therapy [28], acupuncture [29], ultrasound [30], massage [31], spa [32], cupping [33], yoga [34], and laser [35], but there are great differences in the treatment effect on different individuals, and their effect is to relax tense muscles, promote local blood circulation, improve function of the knee joint, and promote absorption and discharge of inflammatory substances.

### 2.2. Drug Treatments

#### 2.2.1. Topical Treatment

Zhao et al. [36] found that oral loxoprofen sodium (LOX-O) was found to be comparable to loxoprofen sodium hydrogel transdermal patch (LOX-T), indicating promising topical use of nonsteroid anti-inflammatory drugs (NSAIDS). Coskun Benlidayi et al. [37] found that both ibuprofen gels and creams had significant clinical efficacy. Wadsworth et al. [38] found that topical administration of 2% sodium diclofenac had not only a good clinical effect, but also, it was well tolerated by patients. Moreover, piroxicam, Tongning gel, also has an obvious curative effect [39, 40]. At the same time, Teymouri et al. [41] found that the bioactive ingredients of herbal gels have obvious healing effects on knee pain, stiffness, and mobility, such as hemp oil, quercetin, *Phyllanthus amarus* Schumach. & Thonn, and Guilu Erxian Glue [40, 42–44].

#### 2.2.2. Oral Treatment

*(1) Nutritional Articular Cartilage*. The European Association for the Osteoporosis and Economic Areas of Osteoarthritis (ESCEO) recommends glucosamine sulfate (GS) and chondroitin sulfate (CS) as first-line treatments for knee osteoarthritis (OA) [45]. Lomonte et al. [46] found that the combination of new glucosamine sulfate and chondroitin sulfate had good efficacy and tolerance. Meanwhile, Lugo et al. [47] found that undenatured type II collagen supplements had good efficacy and be tolerated in regulating symptoms of osteoarthritis in the knee.

*(2) NSAIDs*. NSAIDs (nonsteroidal anti-inflammatory drugs) are the cornerstones of osteoarthritis (OA) therapy, but NSAIDs have gastrointestinal toxicity, while taking gastric mucosal protective agents reduces adverse events in the stomach [48]. In recent years, obvious upper gastrointestinal and cardiovascular adverse events have made rational NSAIDs medication very important. It is recommended that patients with severe symptomatic OA use weak opioids (e.g., tramadol) for a short time. Diacerein, an important inhibitor of new osteoarthritis IL-1, can significantly improve the joint function of patients with osteoarthritis, delay the course of disease, reduce pain, and improve the quality of life of patients [49]. Simental‐Mendía et al. [50] found that the avocado soybean unsaponifiables (ASU) was also beneficial for symptomatic KOA.

*(3) Traditional Chinese Medicine Treatment*. Lai et al. [51] found that in the treatment of knee degenerative osteoarthritis, the 4-week treatment with Duhuo Jisheng decoction can reduce pain and stiffness and improve physical function. Other Chinese patent medicines include Biqi capsule, Fuzheng Guben pill, Xiaohuoluo pill, Gujin pill, Huoxue Zhitong capsule, Jiangu granule, and Xianling Gubao capsule. Furthermore, the herbal formulation combined with conventional treatment appears to be more effective in improving the physiological function of the knee joint [52].

The article "Healthcare and Scientific Treatment of Knee Osteoarthritis" was retracted in 2023. Reasons: signs of a paper mill; compromised peer review; unreliable results or conclusions.

## 3. Surgical Treatment

### 3.1. Intraarticular Puncture and Injection of Knee Joint

Intraarticular puncture and injection of knee joint is an invasive surgical treatment for KOA. Commonly used drugs for puncture and injection include glucocorticoid, ozone, hyaluronic acid, platelet-rich plasma, and mesenchymal stem cells. Intraarticular injection of corticosteroids (IACI) is a common method to relieve pain in patients with knee osteoarthritis (OA). The effective time of intraarticular injection of glucocorticoid is reported to be different, about 1–3 months, while F006, as a new microsphere-based triamcinolone acetonide sustained-release preparation, prolongs the action time [53–56]. The mechanism of ozone may be through activation of the cellular metabolism, reducing prostaglandin synthesis, thereby relieving pain, improving function, and quality of life [57], Intraarticular cavity injection of ozone coupled with oral celecoxib and amino glucose significantly reduced the pain intensity in patients with mild to moderate KOA [58]. Currently, the volume and large variability in the concentration of ozone treatment of KOA exist at the time of injection, so more trials are needed to determine the optimal dose of ozone. Hyaluronic acid (HA) is still in the second-line treatment of NSAIDs in KOA patients, and the benefits are durable compared to IA [59]. Platelet-rich plasma (PRP) is a safe treatment that benefits patients at least in the short term (up to 12 months) and is more effective than HA [60]. Transplanted MSC can differentiate directly into chondrocytes and promote cartilage regeneration, also secreting a range of growth factors and cytokines, where (platelet-derived growth factor) PDGF is the most efficient growth factor and may contribute to tissue integration during cartilage repair or tissue engineering [61, 62]. Early transplantation may yield better results in long-term follow-up [63]. Mesenchymal stem cell therapy may be widely used in the future, as it may confer substantial benefit to patients with KOA.

The article "Healthcare and Scientific Treatment of Knee Osteoarthritis" was retracted in 2023. Reasons: signs of a paper mill; compromised peer review; unreliable results or conclusions.

### 3.2. Knee Arthroscopy

Knee clearing achieved good results in early and middle KOA, and a randomized controlled trial indicated that knee arthroscopic loose lobectomy was more effective than conservative treatment [64]; it can relieve the symptoms for up to 2 years without increasing the risk of joint replacement [65]. In addition, inlay plasty is the replacement of lost cartilage with an autograft harvested from nonload-bearing areas of articular cartilage [66]. Microfracture (MF) prompts the recruitment of pluripotent bone marrow-derived stromal cells to cartilage defects [67]. ACI is an in vitro expansion of autologous chondrocytes harvested from nonload-bearing regions of articular cartilage, then injected into the defect, and covered with a biodegradable collagen membrane [68].

### 3.3. Osteotomy around the Knee

#### 3.3.1. HTO

The biomechanical goal of high tibia osteotomy (HTO) is to readjust the load-bearing line within the coronal plane. The aim was to achieve the transfer of load-bearing lines from the arthritic chamber to a relatively healthy chamber. Pannell et al. [69] found patients treated with HTO have an 8% increased risk of requiring replacement every 1 year, and older, higher rates of complications were more significant in women than in men. HTO can provide long-term survival for certain patients. Patients selected for this surgery should be carefully considered for their age, gender, and osteoarthritis severity.

#### 3.3.2. PFO

Proximal fibular osteotomy (PFO) is a simple and effective method for medial septal OA. Qin et al. [70] performed a proximal fibula osteotomy (PFO) in 52 patients with medial knee OA and varus deformity. The larger distal displacement of the fibula head suggests a greater range of activity in the tibial fibula joint and a more pronounced postoperative improvement in OA symptoms, and proximal bula osteotomy has proven very effective in young patients with medial knee osteoarthritis.

#### 3.3.3. DFO

Distal femur osteotomy (DFO) is a recognized treatment of femoral malformations and associated symptoms (including osteoarthritis). It is commonly used to treat young and physically active patients who do not want a knee replacement. After DFO, 80% of patients could exercise normally and 90% returned to normal work [71]. Shivji et al. [72] retrospectively studied 83 patients with good DFO, results with an average follow-up of 99 months, meaning survival of 113 months (95% CI 106–120), and 89% likelihood of survival of 10 years.

The article "Healthcare and Scientific Treatment of Knee Osteoarthritis" was retracted in 2023. Reasons: signs of a paper mill; compromised peer review; unreliable results or conclusions.

#### 3.3.4. Knee Joint Replacement

*(1) Univentricular Knee Arthroplasty*. Univentricular knee arthroplasty is an operation to protect the bones and preserve ligaments. It has become a lasting and effective method for the treatment of end-stage single compartment KOA. It can effectively reduce postoperative pain and reduce the incidence of postoperative complications [73]. Opioid demand was also reduced when compared to total knee replacement (TKA) [74]. Batailler et al. [75] through studies of robotic-assisted single-cell knee replacement (57 medial and 23 exception side surgeries) found that robotic total knee replacement (TKA) has improved the accuracy of implant positioning and reduced outliers in achieving planned limb alignment [76].

*(2) TKA*. Total knee arthroplasty (TKA) is a new technology for the treatment of knee diseases. The annual incidence of KOA is estimated at 240 per 100,000 patients. About 400,000 initial total knee replacements are done each year in the US. Patient-reported pain and functional outcome scores were significantly improved after successful TKA surgery. Although the overall lifespan of the TKA prosthesis is affected by numerous patients and prosthetic technology-related factors, in all, the average service life is 15–20 years. Clinicians are encouraged to ensure that after all nonsurgical treatments are exhausted, excellent treatment results can be expected in population [77].

## 4. Conclusion

In conclusion, patients with KOA should first choose nonsurgical treatment. If this method fails, the surgical treatment can be selected according to the patient's actual situation. KOA should not use arthroscopic lavage and debridement as routine treatment as only some patients may benefit. Neither method could alter disease progression. ACI or MACI can be used for focal cartilage defect. Osteotomy is recommended for young active KOA patients who are not suitable for joint replacement. Total knee arthroplasty is a safe, economical, and effective method for the treatment of severe knee osteoarthritis. However, relative risks and benefits should be fully considered in treatment. Single compartment knee arthroplasty, HTO, PFO, or DFO can be considered for unilateral severe knee osteoarthritis after considering age, gender, and basic diseases. In conclusion, the treatment of KOA should follow the principle of individualization and step-by-step treatment according to the actual situation of patients, so as to maximize the benefits of patients.

## Data Availability

The data used to support the findings of this study are available from the corresponding author upon request.

The article "Healthcare and Scientific Treatment of Knee Osteoarthritis" was retracted in 2023. Reasons: signs of a paper mill; compromised peer review; unreliable results or conclusions.

## Abbreviations

KOA: Knee osteoarthritis
NGF: Neural growth factor
HIF: Hypoxia-inducible factor
LOX-O: Oral loxoprofen sodium
LOX-T: Loxoprofen sodium hydrogel transdermal patch
NSAIDS: Nonsteroidal anti-inflammatory drugs
ESCEO: Economic areas of osteoarthritis
GS: Glucosamine sulfate
CS: Chondroitin sulfate
OA: Knee osteoarthritis
ASU: Avocado soybean unsaponifiable
IACI: Intraarticular injection of corticosteroids
HA: Hyaluronic acid
PRP: Platelet-rich plasma
PDGF: Platelet-derived growth factor
MF: Microfracture
HTO: High tibia osteotomy
PFO: Proximal fibular osteotomy
DFO: Distal femur osteotomy
TKA: Total knee replacement.
